# Endostatin Inhibits Blood-Retinal Barrier Breakdown in Diabetic Rats by Increasing the Expression of ICAM-1 and VCAM-1 and Decreasing the Expression of VEGF

**DOI:** 10.1155/2022/5105866

**Published:** 2022-01-17

**Authors:** Jinhua Zhou, Zhenggao Xie

**Affiliations:** ^1^Department of Ophthalmology, Yizheng Hospital, Nanjing Drum Tower Hospital Group, Yangzhou 211400, China; ^2^Department of Ophthalmology, Drum Tower Hospital Affiliated to Nanjing University Medical School, Nanjing 210008, China

## Abstract

**Objective:**

Endostatin has become the strongest endogenous angiogenesis inhibitor due to suppressing VEGF expression. The purpose of this study was to assess the impact of endostatin on the blood-retinal barrier (BRB) in diabetic rats.

**Methods:**

SD rats were induced to develop diabetes by streptozotocin, and endostatin was administrated by intravitreal injection. The body weight, the level of blood glucose, the expressions of C-reactive protein (CRP), adhesion molecules intercellular cell adhesion molecule-1 (ICAM-1) and vascular cell adhesion molecule-1 (VCAM-1), junction proteins (occludin, claudin-5, and zonula occluden-1), and VEGF were measured in rats' retinas of diabetes. The BRB breakdown was evaluated using Evans blue.

**Results:**

The level of CRP and adhesion molecules (ICAM-1 and VCAM-1) was increased in retinas of diabetic rats, while endostatin significantly inhibited the upregulation of these. Diabetes increased the BRB permeability and retinal thickness. Diabetes also decreased the levels of occludin, claudin-5, and ZO-1 in retinals. These changes were inhibited by endostatin treatment. Upregulation of vascular endothelial growth factor (VEGF), transforming growth factor-*β* (TGF-*β*), and protein kinase C- (PKC-) *β*2 was also reversed by endostatin in retinas of diabetic rats.

**Conclusions:**

Endostatin provides protection against diabetic retinopathy, which may involve its barrier-enhancing effects.

## 1. Introduction

Diabetic retinopathy is a common and specific microvascular complication of diabetes, and it is still the main cause of blindness prevention among working-aged population [1]. It was found in 1/3 of diabetic patients and is associated with increased risk of life-threatening systemic vascular complications, including stroke, coronary heart disease, and heart failure. Its main pathological change is the destruction of blood-retinal barrier (BRB). The optimal control of blood glucose, blood pressure, and possible blood lipids remains the basis for reducing the risk of retinopathy development and progression [1–3]. Similar to the blood-brain barrier, BRB selectively regulates the microenvironment of retinal nerve tissue, vascular permeability and balance, ion concentration, and transport metabolites [4]. In addition, BRB can limit the immune globulin, albumin, and circulating immune cells into neural retina, which can protect the retinal nerve tissue from the effects of inflammatory cells and cytotoxic in blood [5]. BRB plays an important role in regulating the local microenvironment of the retina and maintaining the homeostasis of retina [6]. BRB destruction is an important part of the pathogenesis of diabetic retinopathy, which can result in increased permeability to lipids and protein and mainly clinically manifested as microangioma, hemorrhage, hard exudation, and macular edema [1, 7].

Vascular endothelial growth factor (VEGF) is a powerful vascular osmotic factor, which can increase the permeability of blood vessels by inducing the phosphorylation of calcadin and close connexin [8, 9]. It has been found that the level of VEGF in vitreous body is significantly elevated in diabetes patients, while the protein and mRNA levels of VEGF in retina are also significantly increased [10, 11]. Highly expression of VEGF under diabetic conditions induced neovascularization and BRB breakdown [12]. These newly formed vessels are more fragile and leaky and more vulnerable to rupture, resulting in more extensive neovascularization, massive bleeding, and loss of vision [13].

Endostatin is one of such antiangiogenic agents currently being studied. It is a carbon terminal protein fragment obtained after cutting the carbon terminal of XVIII collagen [14]. It is one of the most effective angiogenesis inhibitors known at present and is currently undergoing clinical trials [15]. So far, it has been shown to inhibit as many as 65 different types of tumors. In addition, it can also downregulate various pathological types of angiogenesis because of its ability to induce modifications in about 12% of the human genomes. It was reported that Endostar could suppress gastric cancer growth by decreasing the expression of proangiogenic factors, including VEGF and basic fibroblast growth factor (bFGF) in mice [16, 17]. Endostatin is currently undergoing phase II clinical trials and is achieving complete success. It may be approved as an effective drug for antiangiogenesis therapy, considering the application as an angiogenesis inhibitor. However, the role of endostatin in diabetic retinopathy remains to be unknown. Therefore, the present study tried to assess the effectiveness of endostatin on diabetic retinopathy.

## 2. Material and Methods

### 2.1. Animals and Rat Model of Streptozotocin-Induced Diabetes

Ten-week-old male SD rats weigh approximately 200-250 g. Before modeling, fasting blood glucose levels were determined using commercially available enzymatic assays. In addition, glucose tolerance test also was performed. Before the glucose tolerance test, the SD rats were fasted overnight and anesthetized, and then, blood samples were taken. Then, 2 g/kg glucose was intragastric administration. Blood samples were taken, and glucose levels were determined at 30, 60, and 120 min.

Diabetes was induced by an intraperitoneal injection of streptozotocin (STZ; 60 mg/kg in 0.1 mol/L of citrate buffer; Sigma, Shanghai, China) into SD rats. Blood from tail vein was utilized for blood glucose and urine glucose level test after injection 72 h and a week. When rats with blood glucose concentrations higher than 16.7 mmol/L and positive urine glucose, they are considered diabetic rats. The diabetic rats without complications from intravitreal injection (such as retinal detachment, hemorrhages, and infection) were divided into six groups:

- *Group 1: the normal group (n* = 10). The mice were not administrated.
- *Group 2: the STZ group (n* = 10). Diabetic rats did not receive another treatment.
- *Group 3: the low endostatin group (n* = 15). Diabetic rats received intravitreal injection of Endostar (1 *μ*l, 5 mg/ml).
- *Group 4: the middle endostatin group (n* = 15). Diabetic rats received intravitreal injection of Endostar (2.5 *μ*l, 5 mg/ml).
- *Group 5: the high endostatin group (n* = 15). Diabetic rats received intravitreal injection of Endostar (5 *μ*l, 5 mg/ml).
- *Group 6: the positive drug group (n* = 15). Diabetic rats received intravitreal injection of Avastin (2.5 *μ*l, 5 mg/ml).
- *Group 7: the drug combination group (n* = 15). Diabetic rats received intravitreal injection of Endostar (2.5 *μ*l, 5 mg/ml) and Avastin (2.5 *μ*l, 5 mg/ml).

In a separate set of experiments, rats were killed at four weeks in order to collect samples.

### 2.2. Enzyme-Linked Immunosorbent Assay (ELISA)

The concentration of CRP and intercellular cell adhesion molecule-1 (ICAM-1) in serum was determined by ELISA (eBioscience, San Diego, CA) following the manufacturer's instructions. The 96-well microplates were read using a PowerWave X340 microplate reader (Bio-TEK).

### 2.3. Hematoxylin and Eosin Staining and Observation

The retinas were observed by hematoxylin and eosin staining. Briefly, the retinas were fixed in 4% polyoxymethylene, freezed in 30% sucrose, embedded in paraffin, and stained. Slice thickness was set at 5 *μ*m and observed under a microscope. The retinas from each animal were imaged for analysis.

### 2.4. Evans Blue Assay

Evans blue assay was performed to evaluate BRB breakdown. Briefly, Evans blue dye was dissolved in normal saline (30 mg/mL). Then, under anesthesia, the dye (45 mg/kg) was injected through the caudal vein. Blood (200 *μ*L) was withdrawn after Evans blue injection and then every 30 minutes for up to 120 minutes. Then, the chest cavity was opened, and the left heart ventricle was cannulated. Each rat was perfused with citrate buffer (37°C) for 2 min to clear the dye. Immediately after perfusion, eyes were enucleated and the retinas were carefully dissected under an operating microscope. Dry weight is weighed overnight. Evans blue was extracted by incubating each retina in 150 *μ*L formamide (Sigma-Aldrich) for 18 h at 70°C. The supernatant was filtered through centrifugal filter tubes (Millipore, Bedford, MA) at 6000 rp/min for 1.5 h, and 100 *μ*L of the filtrate was used for triplicate spectrophotometric measurements. The background subtracted absorbance was determined by measuring each sample at 620 nm (the absorbance maximum for Evans blue in formamide) and 740 nm (the absorbance minimum). The concentration of dye in the extracts was calculated from a standard curve of Evans blue in formamide. The dry weight of retinas was used to normalize the quantitation of Evans blue leakage.

### 2.5. Western Blotting

Total proteins were extracted from retina tissues using RIPA lysis buffer for 30 min on ice. The loading buffer was added, and mixtures were treated at 100°C for 5 min to denature the protein. Protein concentration was determined by BCA Quantification Kit (Beyotime, Beijing, China). The samples were separated on 10% SDS-PAGE and blotted onto a PVDF membrane. The membranes were blocked with 5% no-fat milk at 25°C for 1 h and incubated with primary antibodies overnight at 4°C. The membrane was incubated with secondary antibody at 25°C for 2 h. The immunoreactivity was visualized using the ECL western blotting kit (Beyotime, Beijing, China) according to the manufacturer's protocols.

### 2.6. Immunofluorescence

Immunofluorescence assay was performed to observe the expression of claudin-5, ICAM, and VEGF. The sections were blocked in PBS with 1% bovine serum albumin and incubated with mouse monoclonal antibody against claudin-5, ICAM, and VEGF (Abcam, Cambridge, MA, USA) overnight at 4°C. Then, a FITC-labeled goat anti-mouse IgG (Beyotime Institute of Biotechnology, Beijing, China) secondary antibody was conducted to detect immunoreactivity. Images were obtained by laser scanning confocal microscopy (Leica, Mannheim, Germany).

### 2.7. Statistical Analysis

All statistical analysis was analyzed by the GraphPad Prism 5 software. Student's *t*-test was applied to compare the difference of two groups. One-way analysis of variance was applied to compare difference between multiple groups. A value of *P* < 0.05 indicated that the difference was statistically significant.

## 3. Results

### 3.1. Effect of Endostatin on Body Weight and Blood Glucose Level

Effect of endostatin on body weight and blood glucose level in STZ-induced diabetic rats is summarized in Table 1. There was a progressive decrease in the body weight and significant increase in blood glucose after STZ administration, while the rats received endostatin or Avastin treatment showed a progressive attenuation of the weight loss induced by STZ, and the level of blood glucose clearly increased (Table 1).

### 3.2. Histological Evaluation

The result revealed that inflammatory cell infiltration in retinal thickness significantly increases due to intraretinal edema in the nerve fiber layer (NFL) and ganglion cell layer (GCL), as well as cell vacuolization in NFL. However, endostatin treatment obviously ameliorated this effect in a dose-dependent way, and the degree of intraretinal edema remarkably reduced. In addition, in Avastin-treated rats, the edema obviously decreased. No histological alteration was observed in the control group rats (Figure 1).

### 3.3. Endostatin Inhibited the Expression of CRP in Serum of Diabetic Rats

C-reaction protein (CRP) is one of the main and sensitive acute phase proteins of human nonspecific inflammatory response, which can cause dysfunction of vascular endothelial cells and eventually lead to retinopathy [18]. ELISA was performed to evaluate the level of CRP in serum. Increased amount of CRP was observed in serum after STZ injection compared to the control group, while endostatin treatment reduced CRP production in a dose-dependent manner (Figure 2).

### 3.4. Endostatin Decreased Blood-Retinal Barrier Breakdown in the Diabetic Retinal

To determine the permeability of the retinal vasculature in diabetic rats and the effect of endostatin on the blood-retinal barrier (BRB) breakdown, we intravenously injected rats with Evans blue albumin. In the diabetic rats, the permeability of BRB was significantly higher than that of the normal group. However, after endostatin treatment, the BRB permeability significantly ameliorated. The BRB permeability of normal rats had no effect (Figure 3).

### 3.5. Endostatin Attenuated the Upregulation of Adhesion Molecules in the Diabetic Rats

The effect of endostatin on the expression of adhesion molecules on the retina tissues, including intercellular adhesion molecule-1 (ICAM-1) and vascular cell adhesion molecule-1 (VCAM-1), was analyzed as shown in Figure 4. The expressions of ICAM-1 and VCAM-1 on the retina tissues significantly increased in diabetic rats compared with normal controls, whereas their expression was significantly decreased in endostatin-treated diabetic rats (Figure 4(a)). Consistent with the results of western blotting, the immunofluorescence assay showed that the level of ICAM-1 on the retina tissues obviously increased in diabetic rats compared to the control, while this level was reversed by endostatin (Figure 4(b)).

In addition, the ELISA revealed an increased amounts of ICAM-1 in serum in STZ-induced rats, while endostatin treatment significantly reduced the increase of ICAM-1 (Figure 4(c)).

### 3.6. Endostatin Prevented the Loss of Junction Proteins in the Diabetic Retinal

To analyze the effect of endostatin on BRB integrity, the expression of tight-junction proteins including zonula occluden-1 (ZO-1), occludin, and claudin-5 was detected by western blotting. As shown in Figure 5, the expressions of ZO-1, occludin, and claudin-5 were significantly decreased in retinas of diabetic rats compared to the control. This decrease was reversed by endostatin treatment (Figure 5(a)). In addition, immunofluorescence assay also revealed a significant reduction in claudin-5 in retinas from STZ-induced rats; however, the endostatin treatment significantly decreased this downregulation (Figure 5(b)).

### 3.7. Endostatin Attenuated the Expression of VEGF

Vascular endothelial growth factor (VEGF) is also involved in the pathogenesis of diabetic retinopathy. Immunofluorescence analysis of retina tissues obtained after STZ administration revealed a positive staining for VEGF. In contrast, less production of VEGF was found in the retina tissues of endostatin-treated rats (Figure 6(a)). In addition, western blotting assay showed that treatment of endostatin significantly inhibited upregulation of VEGF, transforming growth factor- (TGF-) *β*, and protein kinase C- (PKC-) *β*2 in retinas from STZ-induced rats (Figure 6(b)).

## 4. Discussion

Diabetic retinopathy is one of the serious complications of diabetes and has become the most important disease affecting the health [1]. It has been divided into early nonproliferative diabetic retinopathy and later proliferative diabetic retinopathy. The main signs of nonproliferative diabetic retinopathy stage are the disruption of the BRB and exudation increased, resulting in ischemia and hypoxia [19–21]. The mechanism of BRB breakdown has mainly focused on opening the tight junction of retinal vascular endothelial cells and vacuolation of the retinal pigment epithelium and endothelial cell transcytosis [22]. The tight junctions of the retinal vascular endothelial cells are the basis of the structure and function of BRB, which is mainly composed of transmembrane proteins, cytoplasmic attachment proteins, and cytoskeletal proteins, regulating the permeability of BRB [23]. Studies have shown that tight junctions made up of proteins, including ZO-1, occludin, and claudin-5, are important guarantees for the maintenance of the physiological function of BRB [24]. ZO-1, a tight junction-related protein, has been used as an index to observe tight junction barrier function and permeability function of various tissues [9]. In this study, endostatin treatment significantly upregulated the level of ZO-1 in retina tissues of diabetic rats. Occludin is the first discovered transmembrane protein, which is connected with F-actin, maintaining the stability of intercellular connection and permeability of intercellular space [25]. Occludin, the major protein regulating BRB, is located on the tight junction of retinal vascular endothelial cells. Its expression is positively correlated with the permeability of BRB [26]. Our research found that the expression of occludin was significantly decreased in retinas of diabetic rats, but this decrease was reversed by endostatin treatment. Claudin-5 is the main protein that constitutes the tight junction of retinal vascular endothelial cells and is also the main transmembrane protein to form BRB [27]. Our data here revealed a significant reduction in claudin-5 in retinas from STZ-induced rats; however, endostatin treatment could rescue this downregulation.

VEGF, a powerful vascular osmotic factor, is believed to be associated with the destruction of BRB in diabetes [28]. The expression of VEGF is very low in normal physiological condition, while its high expression was found in the pathological condition, such as embryonic period, inflammation, tumor, and diabetes. VEGF derived from retinal Muller cells plays an important role in retinal vascular leakage induced by diabetes and plays a key role in the early retinal inflammation induced by diabetes [29]. In this study, immunofluorescence analysis of retina tissues revealed a positive staining for VEGF after STZ administration. In contrast, less production of VEGF was found in the retina tissues of endostatin-treated rats. In addition, Zhu et al. found that PKC could cause the damage of BRB by regulating VEGF. We found that endostatin could inhibit the expression of PKC-*β*2 induced by STZ from retina tissues.

For malignant murine keratinocytes (PVDA cells), when treated in vivo with Ad-end (adenovirus expressing endostatin gene), an initial proliferation of the endothelial cells into a multilayered surface epithelium was seen but no invasion of the infected cells into the cells of the host was observed, suggesting the inhibitory action of endostatin in the process of angiogenesis. Thus, downregulation of VEGF might be one of the mechanisms by which endostatin works and hence might provide us with a novel approach in the antiangiogenic therapy of diabetic retinopathy [28, 29].

Multiple growth factors, including vascular endothelial growth factor- (VEGF-) A and transforming growth factor- (TGF-) *β*, were upregulated in the diabetic microenvironment, which is vital to the progress of diabetes [30]. In addition, study found that the combination of TGF-*β* and TGF-*β* receptors on retinal vascular endothelial cells increased the basement membrane of capillaries, which lead to lumen stenosis and blood flow changed, resulted in retinal ischemia, hypoxia, and neovascularization in the late stage of diabetic retinopathy [31]. Besides, the hypothesis of the inhibition of NF-*κ*B becomes even stronger due to the results of a research study which concluded that endostatin binds to *α*5*β*1 integrin. It was concluded that endostatin binds to *α*5*β*1 integrin that has been seen in early studies. *α*5*β*1 integrin is a transmembrane integrin receptor, also known as chondrocyte mechanoreceptor, which is responsible for carrying high-intensity mechanical signals [32]. These signals have been confirmed as one of the factors leading to the activation of NF-*κ*B. Therefore, the binding of endostatin to the *α*5*β*1 integrin receptor inhibits the normal physiological signal transduction pathway of the mechanoreceptors of NF-*κ*B, and inhibiting the activation of NF-*κ*B cannot rule out the inhibitory effect on NF-*κ*B activation [32–34].

ICAM-1 and VCAM-1 promoted leukocyte adhesion, caused a release of inflammatory cytokines, growth factor, and vascular permeability factor in vascular endothelial cells, which changes the tight junction of retinal vascular endothelial cells and allows leukocytes to penetrate into the retina [35, 36]. Herein, the expressions of ICAM-1 and VCAM-1 on the retina tissues significantly increased in diabetic rats, whereas their expression was significantly decreased in endostatin-treated diabetic rats.

In summary, endostatin shows a protective effect on diabetic retinopathy in the diabetic rat model. It effectively blocks the increase of VEGF and decrease of ZO-1, occludin, and claudin-5. In addition, angiogenesis is one of the most aggressive features in the pathogenesis of proliferative diabetic retinopathy. Modern therapies are looking for a way to prevent angiogenesis to prevent patients with diabetic retinopathy from eventually becoming blind. Endostatin is an effective molecule used for prevention. It is well known that it is a very effective angiogenesis inhibitor and is currently undergoing clinical trials to determine its role in antiangiogenesis therapy.

## Figures and Tables

**Figure 1:** Histopathology of diabetic retinopathy. Histological evaluation of retina tissues from STZ-injected rats revealed an increased signs of diabetic retinopathy with edema and inflammatory cell infiltration. Treatment with endostatin reduced the degree of diabetic retinopathy.

**Figure 2:** CRP was downregulated by endostatin in serum of diabetic rats. ELISA was performed to evaluate the level of CRP in serum from diabetic rats with different treatments. ^##^*P* < 0.01 vs. the normal group; ^∗∗^*P* < 0.01 vs. the STZ group; ^∗^*P* < 0.05 vs. the STZ group.

**Figure 3:** Endostatin attenuates retinal vascular leakage. (a) Microvascular permeability was assessed by EB staining of retinal whole mounts. (b) Quantification of vascular leakage of EB into the retina. ^##^*P* < 0.01 vs. the normal group; ^∗∗^*P* < 0.01 vs. the STZ group; ^∗^*P* < 0.05 vs. the STZ group.

**Figure 4:** Endostatin attenuated the upregulation of adhesion molecules in the diabetic rats. (a) Western blotting was performed to test the expression of adhesion molecules in the retina tissues from the diabetic rats, including ICAM-1 and VCAM-1. (b) The immunofluorescence assay was conducted to evaluate the expression of ICAM-1 in the retina tissues from the diabetic rats. (c) The level of ICAM-1 in serum was detected by ELISA.

**Figure 5:** Endostatin prevented the loss of junction proteins in the diabetic retinal. (a) Western blotting was performed to test the expression of junction proteins in the retina tissues from the diabetic rats, including ZO-1, occludin, and claudin-5. (b) The immunofluorescence assay was conducted to evaluate the expression of claudin-5 in the retina tissues from the diabetic rats.

**Figure 6:** Endostatin attenuated the expression of VEGF. (a) The immunofluorescence assay was conducted to evaluate the expression of VEGF in the retina tissues from the diabetic rats. (b) Western blotting was performed to test the expression of VEGF, transforming growth factor- (TGF-) *β*, and protein kinase C- (PKC-) *β*2 in the retina tissues from the diabetic rats.

**Table 1:** Blood glucose levels and body weights of STZ-induced diabetic rats.

Groups	*n*	Blood glucose (mmol/L)	Body weight (g)
Normal	10	5.12 ± 1.01	241.12 ± 10.86
STZ	10	26.80 ± 0.48^##^	164.47 ± 19.24^##^
Low endostatin	15	25.40 ± 0.56	168.22 ± 23.14
Middle endostatin	15	21.23 ± 2.58^∗^	183.80 ± 19.21
High endostatin	15	16.23 ± 2.12^∗∗^	198.86 ± 15.23^∗^
Avastin	15	13.21 ± 1.21^∗∗^	200.73 ± 24.66^∗∗^
Avastin+endostatin	15	9.02 ± 0.98^∗∗^	226.05 ± 26.82^∗∗^

Values are means ± SD. ^##^*P* < 0.01 vs. the normal group; ^∗∗^*P* < 0.01 vs. the STZ group; ^∗^*P* < 0.05 vs. the STZ group.

## Data Availability

The data used in this research can be obtained from the corresponding author according to the reasonable requirements.
